The article "Assessing the Contact Angle Between Dentin Treated With Irrigation and Calcium Hydroxide and Root Canal Sealers" was retracted in 2022. Reasons: errors in the data; errors in the methods; errors in the results or conclusions.

# Assessing the Contact Angle Between Dentin Treated With Irrigation and Calcium Hydroxide and Root Canal Sealers

**DOI:** 10.7759/cureus.29474

**Published:** 2022-09-22

**Authors:** Binila S Babu, Nithin Shetty, Nisha C, Noushin Faizal, Mrunalini Vaidya, Nishin K John

**Affiliations:** 1 Department of Conservative Dentistry and Endodontics, Al Azhar Dental College, Thodupuzha, IND; 2 Department of Conservative Dentistry and Endodontics, Ramaiah University of Applied Science, Bangalore, IND; 3 Department of Conservative Dentistry and Endodontics, Ministry of Interior, Doha, QAT; 4 Department of Conservative Dentistry and Endodontics, Dr GD Pol Foundation YMT Dental College, Mumbai, IND

**Keywords:** endodontics, root canal sealers, dentin wettability, chemical irrigation, ca(oh)2

## Abstract

Background

The long-term use of calcium hydroxide, or Ca(OH)2, on dentin has been established in the literature. However, scarce data is available on dentin wettability with Ca(OH)2.

Aim

The present study was conducted to assess the outcomes of Ca(OH)2 use on the wettability of dentin following two and four weeks of using sealers of bioceramic (BC) and Tubli-Seal™ in the root canal.

Methods

In this study, 168 specimens were divided into 12 groups of 14 specimens each and were numbered from G1 to G12. G1-G6 groups were tested with Tubli-Seal. Sterile water irrigation was reserved for G1 for two weeks (14 days) followed by two minutes treatment with 6% sodium hypochlorite (NaOCl) chemical irrigation and 17% EDTA (10 ml). G2 and G3 were subjected to Ca(OH)2 (0.1 ml of UltraCal) for two weeks followed by 10ml sterile water irrigation for two minutes with chemical irrigation. G4 to G6 were given similar treatment for four weeks. G7-G12 were assessed for BC sealer similarly to G1-G6. Two and four weeks of incubation with sterile water or Ca(OH)2 was done in 100% humidity at 37°C. SEM and EDX were done to evaluate the surface morphology of G1 and G6, and results were formed.

Results

Significantly smaller contact angles were seen for Tubli-Seal (G1 to G6) compared to BC (G7 to G12) with p<0.05. Application of water irrigants and Ca(OH)2 (in G2, G5, and G11) showed a smaller (p<0.05, statistically significant) contact angle compared to the use of chemical irrigation agents and Ca(OH)2 (in G3, G6, and G12) except for G8 and G9. Based on EDX and SEM, compared to the use of chemical irrigation with Ca(OH)2, higher remnants of Ca(OH)2 were seen in the water irrigation, whereas, no remnant was seen with chemical irrigants.

Conclusion

Better dentin wettability is seen with Tubli-seal compared to BC sealer. A smaller contact angle between root canal sealers and dentin is seen in the remaining calcium hydroxide samples. Also, calcium hydroxide can be removed from the polished dentin surface with two minutes of irrigation with 17% EDTA and 6% NaOCl.

The article "Assessing the Contact Angle Between Dentin Treated With Irrigation and Calcium Hydroxide and Root Canal Sealers" was retracted in 2022. Reasons: errors in the data; errors in the methods; errors in the results or conclusions.

## Introduction

Ca(OH)2, or calcium hydroxide, has many uses in the field of endodontics including as a root canal sealer and for root fractures, apexification, apexogenesis, intracanal medicament, root resorption, and pulp capping. Non-setting type of Ca(OH)2 is commonly used as a paste mixed with different vehicles for root canal disinfection. The antimicrobial action is imparted hydroxyl ion release raising pH to 12.5, showing the lethal effect on bacterial cells. The role of Ca(OH)2 as an ideal intracanal disinfectant is controversial with different results where few studies report complete eradication of microorganisms after Ca(OH)2 use whereas others reported infection in 26% of cases following Ca(OH)2 use [1]. 

With reported high success rates of using intracanal medicament as calcium hydroxide, adverse effects are reported on long-term use on dentin's mechanical properties making it fracture susceptible. It has been reported that using Ca(OH)2 for four weeks or longer results in decreased mechanical properties and increased fracture susceptibility in in-vitro studies [2]. To get long-term success, preventing communication between periradicular tissues and the oral cavity can be prevented by achieving a three-dimensional (3D) fluid-tight seal which cannot be solely achieved using solid-core root filling materials alone making the use of root canal sealers a vital step. Sealers in root canals are being used to fill gaps and irregularities in the space between the walls of the root canal and the filling materials. Various sealers used in the root canal include calcium phosphate, methacrylate resin-based, calcium silicate phosphate, mineral trioxide aggregate (MTA), silicone, epoxy resin, and zinc oxide-eugenol-based sealers [3].

The most commonly used sealer is zinc-oxide eugenol and epoxy resin based on nearly 74% and 25% endodontic treatments [2]. Tubli-Seal™ is a eugenol-based sealer used in the majority of endodontic practice as it is associated with various advantages including minimal shrinkage of nearly 0.14% compared to resin-based sealers [3]. Additionally, eugenol-based sealers have been shown to have an antibacterial impact on the numerous microorganisms that may be found in a root canal for up to seven days. However, it has the limitation of having the highest solubility compared to other available contemporary sealers [4].

Proper root canal sealer adaptation to the wall is vital to attain a maximum three-dimensional seal while obturating. The wettability and flowability of the root canal sealers can affect the adaptability of sealers to the walls of the root canal. The wetting behavior of any liquid can be accurately indicated by the contact angle [4]. The contact angle of sealers on root canal dentin is affected by the effects on dentin surface tension by various dentin conditions. An evaluation of the contact angle reveals that there is a paucity of information in the scientific literature concerning the wettability of sealers used in the treatment of dentin with Ca(OH)2 [5]. Hence, the present study was conducted to assess the outcomes of Ca(OH)2 use on the wettability of dentin following two and four weeks of using two different sealers in the root canal.

The article "Assessing the Contact Angle Between Dentin Treated With Irrigation and Calcium Hydroxide and Root Canal Sealers" was retracted in 2022. Reasons: errors in the data; errors in the methods; errors in the results or conclusions.

## Materials and methods

The present study was conducted to assess the outcomes of Ca(OH)2 use on the wettability of dentin following two and four weeks of using two different sealers in the root canal. Also, the present study was aimed at assessing the outcomes of applying Ca(OH)2 on the wettability of the dentin following two and four weeks of using the two different sealers in the root canal (ethical approval no: YMTDCH/2021/21/309).

In this study, 168 third molars with no caries were procured and kept at 4°C in the thymol solution (0.1%). Using a saw and constant irrigation, 2 mm sections were made parallel to the crown and close to the pulp. A deep coronal section was used as it provides a wider area. To remove enamel from the sample teeth, silicon carbide paper of 1200-grit was used with water irrigation followed by pulpal side flattening with carbide papers. The specimens were sonicated in deionized water and then placed for three minutes in running deionized water followed by polishing with spray. Then samples were again immersed in running deionized water. For smear layer removal, specimens were treated in 6% NaOCl and 17% EDTA for five minutes. 

These 168 specimens were divided into 12 groups of 14 specimens each and were denoted from G1 to G12. G1-G6 groups were tested with Tubli-Seal. G1 was subjected to irrigation using sterile water for 14 days (two weeks), and then two minutes of chemical irrigation with 6% NaOCl (10ml) and 10 ml of 17% EDTA. G2 and G3 were subjected to Ca(OH)2 (0.1 ml of UltraCal) for two weeks followed by 10ml sterile water irrigation for two minutes/chemical irrigation. G4 to G6 were given similar treatment for four weeks. G7-G12 were assessed for BC sealer similarly to G1-6. Two and four weeks of incubation with sterile water or Ca(OH)2 was done in 100% humidity at 37°C (Figures 1-4).

**Figure 1:** Group 2 subjected to Ca(OH)2 (0.1 ml of UltraCal)

**Figure 2:** Group 3 subjected to Ca(OH)2 (0.1 ml of UltraCal) for two weeks

**Figure 3:** Groups 1-6 tested with Tubli-Seal

**Figure 4:** Groups 7 to 12 assessed for BC sealer BC: bioceramic

The contact angle was measured between calcium silicate-based sealer (BC sealer) or zinc-oxide eugenol-based sealer (Tubli-Seal) and treated dentin surface. These sealers are available in auto mix and premix syringes eliminating manual mixing errors. Before measuring the contact angle, specimens were air-dried for two seconds from a six-inch distance followed by dropping of 2µL sealer drop on dentin. PGX goniometer was used for assessing the contact angle immediately following sealer detachment from the pipette. The contact angle was measured at room temperature in triplicate for each dentin disc.

The article "Assessing the Contact Angle Between Dentin Treated With Irrigation and Calcium Hydroxide and Root Canal Sealers" was retracted in 2022. Reasons: errors in the data; errors in the methods; errors in the results or conclusions.

Also, 18 additional discs of dentin were made and split into six groups (n=3) which were treated similarly and were used for EDX (energy-dispersive X-ray measurement) to assess surface chemical changes following different treatments. Following treatment, samples were dried for 48 hours, and % weight was assessed for nitrogen (N), carbon (C), phosphorus (P), and calcium (Ca) using SEM (scanning electron microscopy). EDX analysis was done on five random spots at X1000 magnification and 15kV. Any remaining Ca(OH)2 and morphological changes in treated dentin surface were assessed on SEM in the 18 samples where they were subjected to a low-vacuum-pressure desiccator for air-drying of each sample for 48 hours. Three scanning electron microscopic images were captured at X1000 magnification for all the samples on the site of the treatment: one from the center, and two from the edges. Cleanliness analysis was done using a 5-grade scale by Alturaiki et al. in 2015 [6].

The collected data were subjected to statistical evaluation using SPSS software version 21 (IBM Corp., Armonk, NY) and one-way ANOVA and t-test for results formulation. The data were expressed in percentage and number, and mean and standard deviation. The level of significance was kept at p<0.05.

## Results

The study results showed that for contact angle, in G1-G6 groups (Tubli-Seal), the highest and lowest contact angle was seen in G4 and G5 with 104.7±6.9° and 85.2±15.3° respectively. In G7-G12 (BC) group, the highest and lowest contact angle was seen for G10 and G11 with 145.2±5.0° and 128.6±8.3° respectively (Table 1).

**Table 1:** Mean contact angle in different study groups

Parameter	Contact angle (Mean±SD)
G1	94.4±11.3
G2	92.4±7.8
G3	98.7±6.8
G4	104.7±6.9
G5	85.2±15.3
G6	99.0±9.4
G7	141.2±4.3
G8	136.9±6.4
G9	130.0±9.6
G10	145.2±5.0
G11	128.6±8.3
G12	142.4±8.4

**Table 2:** Effect of contact angle on various study parameters

Contact angle effects	f-value	p-value
Duration	1.91	0.1668
Type of sealer	922.96	<0.0001
Duration with sealer type	0.33	0.5794
Treatment	20.42	<0.0001
Duration with treatment	12.35	<0.0001
Sealer type with treatment	2.43	0.08
Duration with sealer type and treatment	3.95	0.02

On evaluating the effects of sealer, BC sealer had a significantly higher contact angle compared to Tubli-seal with p<0.0001 (Table 2).

The article "Assessing the Contact Angle Between Dentin Treated With Irrigation and Calcium Hydroxide and Root Canal Sealers" was retracted in 2022. Reasons: errors in the data; errors in the methods; errors in the results or conclusions.

**Table 3:** EDX assessment of 4 elements in different study groups Ca: calcium; N: nitrogen; P: phosphorous; C: carbon

Treatment Type	Duration (weeks)	% Ca (SD)	% P (SD)	% N (SD)	% C (SD)
Chemical (control)	2	0.6 (0.1)	0.4 (0.1)	59.2 (0.2)	39.1 (0.3)
	4	1.1 (0.5)	1.1 (0.2)	57.0 (0.2)	40.3 (1.1)
Ca(OH)2 + water	2	53.4 (2.7)	16.4 (1.2)	18.4 (2.2)	11.0 (0.5)
	4	51.6 (0.6)	17.9 (0.2)	19.0 (0.5)	10.7 (0.2)
Ca(OH)2 + Chemical	2	1.1 (0.1)	1.2 (0.1)	61.2 (2.2)	34.0 (0.2)
	4	3.8 (1.0)	2.7 (0.6)	53.0 (1.0)	35.9 (4.5)

For the Tubli-Seal duration effect, it was seen that G4 had a significantly higher contact angle compared to G1, whereas, a significantly lower contact angle was seen for G5 compared to G2. Between G6 and G3, no significant difference was seen. For BC sealer, at four weeks (G10-12) and two weeks (G7-G9), no significant difference was seen between G10 and G7. A significantly lower contact angle was seen for G11 compared to G8, whereas, G12 had a higher contact angle compared to G9 (p<0.0001). At two weeks for Tubli-Seal, a significantly higher contact angle was seen for G3 compared to G2. Similarly, at four weeks, a higher contact angle was seen for G6 compared to G5. At two weeks for BC sealer, a significantly lower contact angle was seen for G9 compared to G8, and at four weeks, a higher angle was seen for G12 compared to G11 (Table 1). 

For EDX, the measurement of four elements showed a significant assessment of the group, and duration was significant for N. At two and four weeks, the use of water irrigation with calcium hydroxide had significantly higher Ca and P compared to N and C than Ca(OH)2 with chemical irrigation and chemical irrigation without Ca(OH)2. Also, significantly lower C was seen in Ca(OH)2 with chemical treatment compared to chemical irrigation and no Ca(OH)2, and no difference was seen for Ca, P, or N. The two-week similar treatment showed p-values significantly lower compared to four weeks. N was significantly higher at two weeks compared to four weeks. No difference was seen in Ca(OH)2 with water or chemical irrigation. For two and four weeks no significant difference was seen for C in either treatment (Table 2). 

Concerning SEM analysis, effects of treatment duration and groups on calcium hydroxide particle removal were assessed, and it was seen that degree of calcium hydroxide particle removal did not affect the duration. Also, irrigation solution showed a significant effect on calcium hydroxide particle removal and cleanliness with p=0.0006. A higher remnant of calcium hydroxide particles was seen with the water irrigation group compared to chemical irrigation. No remaining Ca(OH)2 following irrigation remained which was the same as seen in the control group (Tables 3-4).

The article "Assessing the Contact Angle Between Dentin Treated With Irrigation and Calcium Hydroxide and Root Canal Sealers" was retracted in 2022. Reasons: errors in the data; errors in the methods; errors in the results or conclusions.

**Table 4:** Assessment of element percentage with duration and treatment type

Treatment	119.44	<0.0001
Duration with treatment	0.16	0.8383

**Table 5:** Alturaiki et al cleanliness scores in study groups

Treatment Type	Duration (weeks)	Scores				
		1	2	3	4	5
Chemical (control)	2	3	0	0	0	0
	4	3	0	0	0	0
Ca(OH)2 + water	2	0	0	2	1	0
	4	0	0	1	1	1
Ca(OH)2 + Chemical	2	3	0	0	0	0
	4	3	0	0	0	0

On assessing the percentage of elements including calcium, phosphorus, nitrogen, and carbon in study specimens, the interaction of duration and group was statistically significant for nitrogen with p=0.01. Also, a statistically significant association was seen for nitrogen with treatment type and duration with treatment type with respective p-values of <0.001 for both. For calcium, a significant association was seen with only treatment type (p<0.0001) and was non-significant for duration and duration with treatment type with p-values of 0.61 and 0.24 respectively. For carbon, a significant association was seen for only treatment type with p<0.001. The percentage of phosphorus in study specimens showed only a statistically significant association with duration and treatment type with respective p-values of 0.03 and <0.0001 respectively as shown in (Table 5).

**Table 6:** Statistical analysis of element percentage, treatment, and duration

S. No	Element and effects	f-value	p-value
1	Calcium		
	Duration with treatment type	1.48	0.24
	Treatment type	1026.84	<0.0001
	Duration	0.22	0.61
2	Phosphorus		
	Duration with treatment type	0.54	0.62
	Treatment type	468.15	<0.0001
	Duration	5.64	0.03
3	Nitrogen		
	Duration with treatment type	5.13	0.02
	Treatment type	505.26	<0.001
	Duration	8.02	0.01
4	Carbon		
	Duration with treatment type	0.16	0.55
	Treatment type	119.44	<0.001
	Duration	0.32	0.55

## Discussion

Obturating the root canals following the biomechanical preparation with the root canal sealers has various proven advantages, including the sealing of the irregularities of the root canal walls like deltas, spaces inaccessible to obturating materials, and the apical ramifications [6]. Root canal sealers also act as binding agents between root canal filling material and the walls of the root canal [7]. Hence, wetting and adequate flow remain the vital physicochemical property of the root canal sealer while obturating. Wettability of the intra-radicular dentin surface largely governs the adhesion of the root canal sealer making contact angle a useful indicator of liquid wettability [8,9].

The article "Assessing the Contact Angle Between Dentin Treated With Irrigation and Calcium Hydroxide and Root Canal Sealers" was retracted in 2022. Reasons: errors in the data; errors in the methods; errors in the results or conclusions.

The contact angle is formed as the tendency exists in a liquid to spread on the surface of the solid surface. When the contact angle is greater than 90^o^, the liquid is considered non-wetting, however, in cases with a contact angle of <90^o^, the liquid is considered as wetting the substrate. Complete wetting is represented by the contact angle of zero. A better interaction is considered between solid and liquid surfaces is considered when the contact angle is low [10,11].

The results of the present study showed that the highest contact angle was seen for the Tubli-Seal group (G1-G6) and the lowest in G4 and G5 with angles of 104.7±6.9^o^ and 85.2±15.3^o^ respectively. For the BC group, the lowest and highest contact angle was seen for G11 and G10 with 128.6±8.3^o^ and 145.2±5.0^o^ angles respectively. Also, Tubli-Seal had a significantly lower contact angle compared to BC sealer (p<0.0001). For duration effects in Tubli-Seal, a significantly lower contact angle was seen in G1 compared to G4, and in G5 than in G2. In comparing G6 with G3, no significant difference was observed. In the groups of BC sealers, no significant difference was seen between G10 and G7. These results were consistent with the findings of Yassen et al. [12] in 2015 and Tummala et al. [13] in 2012 where authors reported comparable contact angle and their effects as in the present study. The lower contact angle of the Tubli-Seal shows that it has better wettability compared to other sealers used in the present study. 

On EDX measurement assessment of duration in the groups was significant for the percentage weight of nitrogen. Significantly lower C and N were seen compared to Ca and P in samples treated with Ca(OH)2 with water irrigation compared to chemical irrigation without calcium hydroxide and chemical irrigation with calcium hydroxide used. Compared to chemical irrigation and no Ca(OH)2, significantly lower C was seen in Ca(OH)2 with chemical treatment with a significantly lower difference at two weeks than four weeks. Lower N was seen at four weeks compared to two weeks. These findings were in agreement with the results of Nagas et al. [14] in 2012 and Mohammadi et al. [15] in 2012 where authors reported similar differences between water and chemical irrigation on dentin wettability. Following EDX, an increase was seen in calcium and phosphate particles. 

After SEM analysis, the effects of treatment duration considered on the removal of calcium hydroxide particles were seen; the duration did not affect the degree of calcium hydroxide particle removal. A significant effect on cleanliness and calcium hydroxide particle removal was shown by irrigation (p=0.0006). Compared to chemical irrigation, in the water irrigation group, more remnants of calcium hydroxide particles were seen. These results were comparable to the studies of Bohn and Ilie [16] in 2014 and Ballal et al. [17] in 2013 where similar SEM findings were seen following the use of calcium hydroxide and different irrigants and removal of remaining particles of calcium hydroxide. SEM analysis showed that following chemical irrigation, calcium particles were not seen irrespective of the treatment duration. However, following irrigation with water, calcium particles were seen.

The article "Assessing the Contact Angle Between Dentin Treated With Irrigation and Calcium Hydroxide and Root Canal Sealers" was retracted in 2022. Reasons: errors in the data; errors in the methods; errors in the results or conclusions.

Study limitations include that this should be evaluated in vivo and hence human-based trials have to be carried out so that other sealer systems can be evaluated. Additionally, this study had a single-assessment time and a smaller number of included samples, thus warranting more long-term studies on a greater number of samples.

## Conclusions

Within its limitations, the present study concludes that better dentin wettability is seen with Tubli-seal compared to BC sealer. The contact angle was lesser between dentin and sealers used in the root canal for the remaining calcium hydroxide samples. Also, calcium hydroxide can be removed from the polished dentin surface with two minutes of irrigation with 17% EDTA and 6% NaOCl. The limitations of the present study were single-assessment time and a smaller number of included samples, warranting more long-term studies on a greater number of samples.
